The article "Concrete Surface Crack Recognition Based on Coordinate Attention Neural Networks" was published in 2022. Journal: Comput Intell Neurosci.

# Concrete Surface Crack Recognition Based on Coordinate Attention Neural Networks

**DOI:** 10.1155/2022/7454746

**Published:** 2022-08-11

**Authors:** Yuhao Zhang, Zhongwei Wang

**Affiliations:** School of Logistics and Transportation, Central South University of Forestry and Technology, Changsha 410004, China

## Abstract

In highway transportation infrastructure such as highways and tunnels, the proportion of concrete consumption is the highest, and concrete cracks are common concrete problems. Concrete cracks will greatly affect the bearing capacity and safety of the structure, easily leading to the interruption of transportation lines, causing great economic losses, and endangering personnel safety. Therefore, the effective identification and timely reporting of concrete cracks is of great significance for the maintenance of infrastructure such as roads and tunnels. In this paper, the CaNet, a deep learning network for identifying concrete cracks, is proposed, which takes ResNet50 as the backbone network. In order to capture the area with a small proportion of cracks, we added coordinate attention to the residual unit of ResNet50 to capture the cross-channel information, direction-aware information, and position-sensitive information from many vertical and horizontal directions so that the network can more accurately locate the narrow crack area. In experiments 3.2 and 3.3, the CaNet has an accuracy rate of 89.6%, which is higher than that of the compared network. In addition, the recall, F1 score, and precision of the CaNet network are 86%, 85%, and 87% , respectively. Therefore, the CaNet model is effective for identifying concrete cracks.

## 1. Introduction

The rapid take-off of the world economy benefits from the stable and sustainable development of the transportation industry to a certain extent. Highways and tunnels are the carriers of the land transportation industry [1], and their structure directly affects whether the transportation lines can continue to operate. However, with the increase in operation time of highway and tunnel facilities and the influence of external environmental factors, certain damage will inevitably occur to highway and tunnel engineering structures [2, 3]. To maintain the normal operation of the transport lines, the transportation department needs to continue the health inspection of highways and tunnels regularly. In highway and tunnel engineering structures, the proportion of concrete consumption is the highest, and shrinkage cracks, broken plates, and ash will cause concrete quality defects, which will not only affect the overall beauty but also affect the quality of the highway and tunnel [4]. Among them, shrinkage concrete cracks are common concrete problems, which are manifested in the process of condensation. If the water evaporates quickly, it will indicate that it is easy to shrink, thus forming irregular or penetrating cracks [5]. The occurrence of cracks will not only reduce the impermeability of buildings but also affect the use function of buildings, causing corrosion of reinforcement, carbonation of concrete, and reducing the durability of materials, Finally, it will affect the bearing capacity of the building. Therefore, timely and effective detection of highway and tunnel surface cracks, detection of possible safety problems, and repair can effectively prevent accidents [6].

The article "Concrete Surface Crack Recognition Based on Coordinate Attention Neural Networks" was published in 2022. Journal: Comput Intell Neurosci.

In real life, manual patrol inspection is still used for the patrol inspection and maintenance of cracks on the surface of highways and tunnels, relying on close observation with the help of width measuring instruments, tape, and other measuring instruments to complete the collection of crack information and mark and record the crack information in time [7]. However, manual patrol inspection has many disadvantages: (1) manual patrol inspection is easily disturbed by human subjective factors and is subject to the experience of patrol inspectors. (2) The safety of personnel cannot be effectively guaranteed when the crack at the high position is inspected, or the detection position is in a relatively steep place. (3) With the development of the world economy, the number of roads, tunnels, and other infrastructure is increasing day by day. If the manual inspection method is adopted, it will cause a lot of waste of human, material, and financial resources. Moreover, the recorded data information is manually recorded, making it difficult to form a complete database, cannot be preserved for a long time, and cannot be comprehensively analyzed with big data technology. As a result, the transportation department must still figure out how to complete concrete surface detection quickly and accurately [8].

To solve the problems encountered in manual inspection, the traditional digital image processing technology for concrete cracks is widely used [9]. For example, Talab et al. [10] proposed a method to identify cracks in concrete images by taking advantage of the characteristics that cracks are dark areas in the image that have a large gap with the background. First, Sobel is used to extract the edges of grayscale images. The foreground and background of all pixels are separated by the threshold method; then, the Sobel or median filter is used to eliminate residual noise. Finally, the Otsu method is used for crack detection. However, the method based on edge detection is easily disturbed by the background information, and it is difficult to recognize the crack features in the image under a complex background. In order to reduce the influence of background on recognition, Shi et al. [11] used the random structured forest method to realize the image detection of complex road cracks, which to some extent solved the problem of difficult recognition under complex background, but the effect was not significant enough. Although the above processing methods have achieved good recognition results, the feature extractor is extremely dependent on the professional knowledge and design experience of designers, and the designed algorithm is only effective in the characteristic scene with low generalization.

The article "Concrete Surface Crack Recognition Based on Coordinate Attention Neural Networks" was published in 2022. Journal: Comput Intell Neurosci.

Compared with the traditional digital image processing technology, the extensive promotion of deep learning has greatly improved the ability of concrete crack feature extraction and feature expression [12]. At the same time, by using a large amount of data for end-to-end self-learning, they can solve well the problem of insufficient generalization. Cha et al. [13] combined the SWT with CNN to detect concrete cracks, which can scan any crack greater than a 256 × 256 resolution image. Experiments show that the method combined with SWT and CNN has better performance in concrete crack identification than the Canny and Sobel detection methods, and the recording accuracy is about 98%; pan et al. [14] developed a layered network called SCHNet, which is composed of the VGG19 backbone network and a self-attention mechanism, and can support pixel-level automatic and reliable concrete crack segmentation. Experiments show that the average IOU reaches 85.31%. Wang et al. [15] used the improved inception RESNET V2 model to identify bridge cracks. The experimental results show that each performance index has been improved to varying degrees: the accuracy is 99.24%; the recall rate is 99.03%; fF-measure is 98.79%; FPS is 196. Nayyeri and Zhou [16] based the MR-CrackNet model to identify cracks of different sizes in roads and bridge decks, and trained and tested it on a new crack dataset containing 2,532 concrete crack images. The experimental results show that MR-CrackNet is superior to the baseline model and can achieve high-precision crack identification. In this paper, the structural features of concrete cracks are extracted by designing the deep learning network structure to distinguish whether the concrete in the image has cracks.

Based on ResNet50 in the ResNet series [17] as the backbone network and adding coordinate attention to the residual unit, this paper proposes CaNet. Coordinate Attention (CA) [18] considers the location information of concrete cracks through the vertical and horizontal characteristic directions and models the long-term dependence so as to enhance the weight of the crack area and distinguish it from useless information such as background.

The article "Concrete Surface Crack Recognition Based on Coordinate Attention Neural Networks" was published in 2022. Journal: Comput Intell Neurosci.

The main contributions of this paper are as follows:

1. The CaNet is proposed: coordinate attention is introduced, which enhances the extraction of micro features of concrete cracks and improves the recognition accuracy of crack images by 6.2% to ResNet50.
2. Compared with several neural networks set up in the experiment, the CaNet has a higher recognition rate in the identification of concrete cracks.

In the second section, we introduced the dataset (2.1) used in this paper and the constituent elements of the CaNet (2.2); the third chapter introduces the experiment performed in this paper, in which 3.1 describes the hardware and software configured for this experiment; 3.2 tests the practicality of the model; 3.3 tests the effectiveness of coordinated attention; 3.4 tests the comparison with other models. The fourth chapter introduces the conclusions and shortcomings of this paper.

## 2. Materials and Methods

### 2.1. Data Acquisition

The quality of the concrete crack dataset can greatly affect the designed network [19, 20]. This time, the concrete crack data set is from Kaggle's surface crack detection public data set [21]. The public dataset has 40000 images, all of which are RGB channels, 227 × 227 pixels, including 20000 images without cracks and 20000 images with cracks. Some images are shown in Figure 1. At the same time, when examining the dataset, it is found that the high-resolution images have great differences in surface finish and lighting conditions, as shown in Figure 2.

### 2.2. Concrete Crack Identification Based on CaNet Model

In CaNet, the main structure of ResNet50 is used. On each floor, 1 × 1 and 3 × 3, coordinate attention is added between convolution blocks. The network structure of CaNet is shown in Figure 3.

#### 2.2.1. ResNet50 Model

In the field of recognising concrete crack images, the depth convolution neural network has produced ideal results recently [22]. The amount of image information that the deep convolution network can learn increases with the number of network layers [23]. However, as the number of network layers rises, over-fitting and network model degradation issues will also arise, making it more difficult to train models and preventing the system from convergence. He K and others [15] created a residual block by incorporating shortcut connections into the original DCNN [24] network structure (RB).  Figure 4 depicts the RB structure.

ResNet50 is a network structure commonly used in various fields, which is formed by stacking different residual blocks. Residual block (RB) is shown in formula :

(1) $$\begin{array}{c} H=F\left(x,\left\{W\right\}\right)+x, \end{array}$$

*x* represents the input characteristic diagram of RB; *H* represents the output characteristic diagram of RB; *F*(*x*, {*W*}) represents the residual mapping of the network. The dimension of input *x* must be the same. If the dimension is different, *W*_*q*_ linear projection should not be added to the shortcut connection, as shown in the following formula:

(2) $$\begin{array}{c} H=F\left(x,\left\{W\right\}\right)+Q\left(x,\left\{W_{q}\right\}\right)\text{.} \end{array}$$

The article "Concrete Surface Crack Recognition Based on Coordinate Attention Neural Networks" was published in 2022. Journal: Comput Intell Neurosci.

#### 2.2.2. Coordinate Attention

The 2D global pool is used to calculate channel attention in the most widely used squeeze and stimulate (SE) attention mechanism. However, SE only takes into account the coding of information between crack channels for concrete crack images, ignoring the significance of concrete crack location data, which is crucial for capturing the object structure in concrete crack recognition. Using the convolution layer to calculate the spatial attention information of concrete cracks, BAM [25] and CBAM [26] attempt to build the crack location information based on the SE attention mechanism's weakness. The long-term dependency required in computer vision tasks cannot be established by convolution though.

In order to address this issue, Hou et al. [18] suggested coordinate attention, which combines the vertical and horizontal inputs into two distinct directional graphs. The location data for cracks are then encoded into two crack attention maps from two-directional maps with different directions of cracks. This allows the generated crack attention map to store the location data for cracks. In order to emphasise the expression of interest, the two crack attention maps are finally applied to the input through multiplication.  Figure 5 illustrates the precise organisation of coordinate attention.

Specific implementation process is

**Step 1 .**

Each channel of input *X* is encoded using a pooling kernel of size (*H*,  1) or (1,  *W*), respectively.

The crack features output of *c* channel with *h* height can be expressed as

(3) $$\begin{array}{c} z_{C}^{h}\left(h\right)=\frac{1}{W}\sum_{0\leq i<w}x_{C}\left(h,i\right). \end{array}$$

The crack features output of *c* channel with *w* width can be expressed as

(4) $$\begin{array}{c} z_{C}^{w}\left(w\right)=\frac{1}{H}\sum_{0\leq j<H}x_{C}\left(j,w\right). \end{array}$$

**Step 2 .**

After the transformation in information embedding, this part concatenates the feature map after step 1 transformation and then uses the convolution to transform it.

(5) $$\begin{array}{c} f=\delta \;\left(F_{1}\left(\left[z^{h},z^{w}\right]\right)\right), \end{array}$$

where *F*_1_ stands for 1 × 1 convolution kernel; *δ* indicates nonlinear activation function; *f* ∈ *ℝ*^*C*/*r*×(*H*+*W*)^ represents the intermediate feature map for coding the spatial information of cracks, and *r* represents the reduction rate of control block size.

The article "Concrete Surface Crack Recognition Based on Coordinate Attention Neural Networks" was published in 2022. Journal: Comput Intell Neurosci.

**Step 3 .**

Divide *f* ∈ *ℝ*^*C*/*r*×(*H*+*W*)^ in step 2 into *f*^*h*^ ∈ ℝ^*C*/*r*×*H*^ and *f*^*w*^ ∈ ℝ^*C*/*r*×*W*^. Then, use 1 × 1 convolution kernels to transform *f*^*h*^ and *f*^*w*^.

(6) $$\begin{array}{c} g^{h}=\sigma \left(F_{h}\left(f^{h}\right)\right),\\ g^{w}=\sigma \left(F_{w}\left(f^{w}\right)\right). \end{array}$$

*σ* stands for the sigmoid function. Both *F*_*h*_ and *F*_*w*_ represent 1 × 1 convolution. *g*^*h*^ and *g*^*w*^ represent weight characteristics.

**Step 4 .**

Use multiplication to fuse weights *g*^*h*^ and *g*^*w*^ with input *X* and output coordinate attention block *Y*, as shown in the following equation.

(7) $$\begin{array}{c} y_{C}\left(i,j\right)=x_{C}\left(i,j\right)\times g_{C}^{h}\left(i\right)\times g_{C}^{w}\left(j\right). \end{array}$$

## 3. Results and Analysis

### 3.1. Experimental Environment and Setting

In this experiment, the network training and testing environments were carried out on a platform. The experimental parameters of training and testing are shown in Table 1.

The concrete crack dataset used this time is the Surface Crack Detection public dataset with 40000 images, which are divided into two types, crack free images and crack images. In all experiments of this paper, according to the ratio of 7 : 2 : 1, the dataset will be divided into the training set, test set, and verification set.

### 3.2. Application Scenarios

Concrete is indispensable in today's construction projects and is the most widely used building material. It is widely used in the construction of infrastructure such as roads, bridges, housing construction, tunnels, and dams. Concrete cracks are the most common quality problem in concrete subprojects. Due to the low tensile strength of concrete and the combined effects of internal and external influences, such as shrinkage and creep, external temperature changes, and foundation deformation, concrete in construction and operation is used. Structures often have cracks to varying degrees and forms, and it is still impossible to completely prevent and eliminate them. Therefore, efficient inspection and monitoring of concrete cracks have become the key to ensuring the quality of concrete projects. Accurately identifying the length, direction, and width of cracks in concrete structures plays an important role in judging the disease degree and operating conditions of the structure.

The article "Concrete Surface Crack Recognition Based on Coordinate Attention Neural Networks" was published in 2022. Journal: Comput Intell Neurosci.

Surface-based crack identification is a considerable task in health monitoring of structures. If cracks continue to expand, they will reduce the effective bearing surface area and can lead to structural failure over time. On the one hand, the detection process of manual cracks is time-consuming and labor-intensive, subject to the subjective judgment of inspectors, and for high-rise buildings and bridges, due to the large operational limitations, manual inspection may also be difficult to perform. On the other hand, although the image recognition technology of AI has been improved dramatically, and the technology of automatically detecting cracks through image recognition has been developed, most of them still require manual image acquisition work, and a lot of high-resolution image data are obtained, but it still takes a considerable amount of time and cost to record the crack detection and make the result file. Therefore, in this paper, we build a convenient and accurate crack identification model based on coordinate attention and test the model on real-world data (the recognition process is shown in Figure 6) and find that the model detects concrete and nonconcrete structure example roads that are accurate in terms of surface cracks. The results of experiment 3.3 show that the target recognition speed and accuracy of concrete surface crack detection technology based on coordinate attention can meet the requirements of real time. It has been widely used in the automatic identification of structural cracks in concrete structures of roads, bridges, and dams and has achieved good practical application results. However, there are still some problems to be solved in the application of the actual scene of structural crack detection, especially for some situations where the on-site detection environment is more complicated, such as water stains on the concrete surface, climbing vines, artificial painting marks, expansion joints, and so on. The structural cracks cannot be accurately identified.

With the continuous improvement of Internet technology and the support of related hardware, artificial intelligence technology has developed rapidly, and it also provides a foundation for big data processing and application. At the same time, the popularity of smart phones, intelligent unmanned aircraft, and intelligent robots has also provided great convenience for big data collection. Based on this, this paper proposes to combine artificial intelligence with project engineering management; use artificial intelligence to collect concrete crack pictures; then use the artificial intelligence coordinate attention neural network to identify and locate cracks in pictures to achieve the purpose of crack detection and monitoring. Making full use of the advantages of artificial intelligence technology makes it possible to collect big data of concrete crack pictures and detect cracks. In addition, we deploy the trained CaNet model to the flask back-end framework and use the uni-app front-end writing framework to design the user interface, thus completing a landing project. At the same time, we used our smartphone to photograph cracks and crack-like noises from surrounding buildings and roads. A total of 100 cracked and uncracked images were taken with a resolution of 4000 × 1800. The configuration of the mobile phone is shown in Table 2, and some pictures are shown in Figure 7.

The article "Concrete Surface Crack Recognition Based on Coordinate Attention Neural Networks" was published in 2022. Journal: Comput Intell Neurosci.

We successively input the captured pictures into the CaNet model for testing and repeat the process to other networks for comparison. The recognition results are shown in Table 3.  Table 4 shows the running smart phone configurations.

### 3.3. Effectiveness Experiment of Coordinate Attention

To test the effectiveness of coordinate attention in the CaNet and determine its improvement on mAP and accuracy, we used SE, CBAM, and CA attention mechanisms as single variables in the experiment, and the invariant was the basic network ResNet50. The results of attention mechanism networks comparison are shown in Table 5.

It can be seen from Table 1 that the three attention mechanisms can improve the map and accuracy. Among them, CA can improve the mAP and accuracy of the network.

### 3.4. Comparison with Other Networks

We compare CaNet with other networks in concrete crack identification and prove that its performance in concrete crack identification is better than other models. In this comparative experiment, we have compared 7 kinds of deep learning networks. The results of network comparison are shown in Table 6.

## 4. Conclusion

In this paper, we construct CaNet to identify concrete cracks. In experiment 3.2, we have tested the recognition effects of CNN, ResNet50, and CaNet on concrete cracks in practical applications. The performance indexes of CaNet we proposed are better than the other two models. In experiment 3.3, we compared the effectiveness of the three attention mechanisms and concluded that coordinated attention improved the network the most in mAP and accuracy, by 8.7% and 6.2%, respectively. In experiment 3.4, we tested the performance of several groups of deep neural networks for concrete crack detection. The recall, F1-score, and precision of CaNet are 86%, 85%, and 87%, respectively, which are better than other networks. These experiments show that the CaNet model is effective for identifying concrete cracks, but further research is still needed. (1) At present, the focus of the research is to identify the concrete crack images of highways and tunnels to complete the classification task. Later, it can be extended to the detection task of wall cracks and metal cracks. (2) The data in this network training are all from the public dataset. In the future, cameras, smartphones, and other shooting equipment should be used to collect concrete crack images in different scenes, expand the dataset, and improve the generalization of the model.

The article "Concrete Surface Crack Recognition Based on Coordinate Attention Neural Networks" was published in 2022. Journal: Comput Intell Neurosci.

## Figures and Tables

**Figure 1:** Partial image display.

**Figure 2:** Partial image difference.

**Figure 3:** The overall architecture of CaNet.

**Figure 4:** Residual block.

**Figure 5:** Coordinate attention.

**Figure 6:** Training and recognition process of the concrete crack recognition model.

**Figure 7:** Take some pictures.

**Table 1:** Experimental parameters of CaNet.

Parameter type	Parameter name	Parameter setting
*Hardware environment*	Operating system	Windows 10 (64 bit)
	Version number	20H2
	RAM	64 GB(63.8 available)
	Processor	Intel(R) core(TM) i7-9700u
	Graphics card	2080ti GPU

*Software environment*	CaNet	Python 3.8.12
		Pytorch 1.8.2
		CUDA 10.2

*Training parameter setting*	Batch size(training)	32
	Batch size(testing)	8
	Learning rate *lr*	10^−3^
	Epoches	140
	Optimizer	Adam optimizer
	Loss function	Cross entropy loss
	Training method	Incremental gradient descent

**Table 2:** Camera phone configuration.

Mobile phone configuration	Value
Processor	Qualcomm snapdragon 870 eight core
Running memory	8.00 GB
Operating system	Android 12
GPU	Adreno 650
Rear camera	71million pixels

**Table 3:** Actual test results.

Network model	Recall (%)	*F*1-score (%)	Precision (%)	mAP (%)	Accuracy (%)
CaNet	82	83	84	83	87
CNN	71	69	75	73	76
ResNet50	79	75	77	75	79

**Table 4:** Operating environment.

Mobile phone configuration	Value
Processor	Qualcomm snapdragon 870 eight core
Running memory	8.00 GB
Operating system	Android 12
GPU	Adreno 650

**Table 5:** Comparison of attention mechanism networks.

Network model	mAP (%)	Accuracy (%)
ResNet50	77.1	83.4
ResNet50-SE	79.7	85.3
ResNet50-CBAM	83.5	87.7
CaNet	85.8	89.6

**Table 6:** Results of comparative experiments.

Network model	Recall (%)	*F*1-score (%)	Precision (%)
DCNN [22]	76	73	77
ResNet50 [15]	79	76	79
SENet [23]	81	79	82
ResNet50-BAM [24]	84	82	83
ResNet50-CBAM [25]	84	80	85
SCHNet [14]	85	84	84
CaNet	86	85	87

## Data Availability

The dataset can be found here: https://www.kaggle.com/datasets/arunrk7/surface-crack-detection?resource=download.
